The article "Economic Transformation and Security Analysis of RMB Integration Based on CNN" was published in 2022. Journal: Comput Intell Neurosci.

# Economic Transformation and Security Analysis of RMB Integration Based on CNN

**DOI:** 10.1155/2022/6732087

**Published:** 2022-07-31

**Authors:** Liming Gong

**Affiliations:** School of Finance, Xi'an Eurasia University, Xi'an, Shaanxi 710065, China

## Abstract

Due to the productivity shocks, there exist inherently systemic biases when using purchasing power parity as the equilibrium real exchange rate measure standard. In this paper, based on the characteristic of Chinese economic transformation, considering demographic and weakened Balassa–Samuelson effect, we reestimate the equilibrium level of the real exchange rate of RMB with the quarterly frequency data since 1994 and measure the misalignment of the RMB real exchange rate. The empirical results show that the improved convolutional neural network (CNN) model is a reasonable analytical framework for the RMB equilibrium real exchange rate, and in the sample period, the real exchange rate of RMB is robust, and demographic is an important variable affecting the RMB equilibrium exchange rate. The real exchange rate of RMB is closely related to China's economic development strategy.

## 1. Introduction

Since the people's bank of China implemented a managed floating exchange rate system for the RMB exchange rate in January 1994, many western countries have criticized China's manipulation of the exchange rate. The US Treasury Department has proposed several bills to the congress to label China as a “currency manipulator.” At present, the RMB has been included in the SDR and has been pegged to a basket of currencies instead of the US dollar. The trading range of the RMB against the US dollar has been expanded to 2%, and the RMB has really evolved into a managed floating exchange rate system determined by the market. The internationalization of RMB requires a strong exchange rate and strong purchasing power. In 2017, the trade dispute initiated by the Trump administration on China made scholars discuss whether the RMB exchange rate should be devalued to deal with trade barriers. All these problems need to determine the equilibrium level and dislocation of the RMB exchange rate.

## 2. Relevant Knowledge

### 2.1. Neural Network Model

With the development of productive forces and the globalization of finance, economic exchanges among countries in the world are becoming more and more frequent, so as to further promote the integration of the global economy. Because of the internationalization of world finance, the depth and breadth of financial penetration are more obvious and prominent. The fluctuation of foreign exchange rate not only has an impact on national financial relations but also affects the economic development of many fields in various countries and plays a more and more important role. Uusivuori et al. [1] studied the exchange rates of currencies of different countries against the US dollar. Through comparative analysis, he found that the exchange rates of these countries were different and finally determined that GARCH (1, 1) model had high prediction accuracy. Cerisola [2] used the autoregressive model to study foreign exchange. The results showed that the average percentage error-index value of the prediction result of the AR (1, 1) model was lower than that of the ARMA (1, 1) model. Based on the research results, it was confirmed that the AR model can significantly improve the accuracy of foreign exchange rate prediction. Chen [3] used the GARCH model and ARIMA model to model the historical data of RMB against the US dollar. Through comparative analysis, the GARCH model has a good performance in the historical data of RMB against the US dollar. Amjady and Ehsan [4] tried to use an artificial neural network to predict the foreign exchange market. According to the conventional method of machine learning, the data are divided into training data and test data. The test data are used as the final verification data set. The results show that artificial neural network has obvious advantages in predicting foreign exchange rate compared with previous research methods. Gevrey et al. [5] successfully used artificial intelligence to solve the interest rate problem between multiple exchange rates and established relevant models to provide relevant support for financial market investment. In order to predict the short-term fluctuation of the exchange rate between the mark and the US dollar, McGroarty et al. [6] used the transaction data in the foreign exchange market in New York and London for modeling and analysis. The prediction results show that the prediction accuracy of the neural network is higher than that of the traditional prediction model. Chai et al. [7] used a genetic algorithm to optimize BP neural network and used the optimized model to predict the exchange rate of RMB against the US dollar. The results show that the neural network model has achieved good results in exchange rate prediction. Sivri et al. [8] have shown that when using the combined model of AR model and ANNs model for exchange rate prediction, the prediction result of the combined model is better than that of the ARIMA model alone. Wu [9] used the ARIMA-NN model to predict the RMB exchange rate. The results show that the prediction accuracy of the ARIMA-NN hybrid model is higher than that of the random walk model, ARIMA model, or NN model. Hirasawa et al. [10] proposed an improved convolutional neural network (CNN) using the deep learning method to establish the short-term model and long-term model, respectively, for the prediction of exchange rate fluctuations. The results show that media indicators can improve the prediction ability of the model in the short-term model. The prediction result of the combination of the short-term model and long-term model is better than that of modeling directly using all influencing factors. Liu et al. [11] mixed the SVR model and ARIMA model to predict the exchange rate of four currencies against the US dollar. The time series of the foreign exchange rate is divided into linear time series and nonlinear time series. ARIMA model is used to predict the linear part of the foreign exchange rate, and the SVR model is used to predict the nonlinear part of the foreign exchange rate.

The article "Economic Transformation and Security Analysis of RMB Integration Based on CNN" was published in 2022. Journal: Comput Intell Neurosci.

### 2.2. Country-Specific Fixed Effects

Due to the impact of productivity factors, the real exchange rate of catch-up economies tends to be underestimated compared with that of developed economies. The Balassa–Samuelson effect (later referred to as the BS effect) provides an analytical framework for studying the impact of productivity shocks on a country's real exchange rate. In recent literature, some scholars estimated the equilibrium real exchange rate of RMB by using the extended PPP model (adding BS effect and other influence factors on the basis of traditional PPP) [12, 13]. From the perspective of high-frequency time series, some scholars have reselected variables affecting the real exchange rate and made some innovations [14, 15].

### 2.3. Population, Exchange Rate, and Balassa–Samuelson Effect

The change in the real exchange rate will be affected by different impact factors, and the transmission mechanism of different impact sources is also different. Considering that the currency is neutral in the long run when analyzing the long-term trend of the real exchange rate, the impact of the real shock on the real exchange rate is mainly investigated. Productivity impact is the main influencing factor. Balassa–Samuelson effect provides an analytical framework for studying the impact of productivity shocks on a country's real exchange rate. The transmission mechanism of Balassa–Samuelson effect is assuming that the traded goods satisfy the one price theorem, the prices of the traded goods of the two countries will converge, and the difference in the productivity level of the tradable sectors of the two countries will determine their wage rate difference, and the faster the productivity growth, the higher the wage level. If the labor force flows freely in China, the wage rates of the two sectors in the economy will converge, but the productivity of the nontradable sector is less than that of the tradable sector, and since the price level is mainly determined by the wage level, the price level of nontradable goods will be higher than that of tradable goods, and at this time, the real exchange rate of the country will appreciate.

The article "Economic Transformation and Security Analysis of RMB Integration Based on CNN" was published in 2022. Journal: Comput Intell Neurosci.

As for the actual situation in China, the classical assumption of full employment due to the limited labor supply in Balassa–Samuelson effect is quite different from the situation in China. Due to the existence of urban-rural dual structure in China's economy and hidden unemployment in rural areas, the labor force is not fully employed, and at the same time, due to the factors of structural transformation, the labor force will be almost equivalent to unlimited supply in a certain period of time. These factors will restrain the increase in the wage rate to some extent.

As can be seen from Figure 1(a), in most years since the reform of the exchange rate system, the annual growth rate of labor productivity in China's manufacturing and service industries has been higher than that in the United States over the same period, and at the same time, as the core transmission mechanism of Balassa–Samuelson effect, the annual growth rate of China's manufacturing productivity is much higher than that of the United States in the same period.  Figure 1(b) shows the trend of China-US relative productivity (cpzs) and RMB real effective exchange rate (REER), when cpzs rises, REER also rises, and vice versa. These characteristics meet the description of Balassa–Samuelson effect. The most important point in the transmission mechanism of Balassa–Samuelson effect is that when the labor productivity of tradable sectors increases relative to that of nontradable sectors, the wage rate also increases correspondingly. If there is a difference between the wage rate and productivity growth in tradable sectors, it indicates that other factors (such as demographic factors) hinder the transmission between them.  Figure 1(c) shows the cumulative growth index of China's manufacturing productivity and its wage rate, and after the reform of the exchange rate system, the labor productivity of China's manufacturing industry has increased by 743%, while the wage rate of this sector has only increased by 456%.

### 2.4. Traditional Research Methods and Advantages of CNN

The financial market can reflect the operation of economy and enterprises. In general, the traditional analysis method is to predict the future development through the current situation of social economy and enterprise development. There are two mainstream traditional analysis methods: event-driven analysis method and performance-driven analysis method as shown in Table 1.

The article "Economic Transformation and Security Analysis of RMB Integration Based on CNN" was published in 2022. Journal: Comput Intell Neurosci.

The computer-based research method takes the algorithm as the core to process and analyzes the data in time, the convolutional neural network adopts an “end-to-end” idea, and the whole prediction process does not carry out the artificial division of subproblem; instead, the convolution neural network(CNN) model is used to realize the transformation from the original input to the desired output, and based on this idea, synergy can be realized and can get the global optimal solution of prediction under the condition of greater possibility.

### 2.5. ICNN and Balassa–Samuelson Effect of RMB Equilibrium Exchange Rate

There are many problems in the traditional econometric modeling theory. Combined with the latest achievements of current econometrics, first, an unstructured method is introduced to establish the relationship model between economic variables, namely vector autoregressive model (VAR). The model is divided into two types, namely nonrestrictive VAR and restrictive VAR. Suppose that *e*_*t*_ = (*e*_1*t*_, *e*_2*t*_,…, *e*_*mt*_)′ represents an *m* dimensional random time series, *q* represents the lag order of the series, and *c*_*t*_ = (*c*_1*t*_, *c*_2*t*_,…, *c*_*mt*_)′, which is an *m* dimensional random disturbance time series. Under nonlimiting conditions, it can be expressed as

(1) $$\begin{array}{c} e_{t}=D_{1}e_{t-1}+D_{2}e_{t-2}+\cdots +D_{q}e_{t-q}+c_{t},\;t=1,2,\ldots ,T. \end{array}$$

Furthermore, if the lag operator is introduced, it can be expressed as

(2) $$\begin{array}{c} D\left(U\right)e_{t}=c_{t},\;t=1,2,\ldots ,T\\ D\left(U\right)=I_{m}-D_{1}U-D_{2}U^{2}-\cdots -D_{q}U^{q}, \end{array}$$

where *D* (*U*) represents the polynomial of lag operator.

Under restrictive conditions, *e*_*t*_ is regarded as an *m* dimensional endogenous random time series, which is affected by the *b* dimensional exogenous time series *f*_*t*_ = (*f*_1*t*_, *f*_2*t*_,…, *f*_*mt*_)′, and correspondingly, VAR can be expressed as

(3) $$\begin{array}{c} e_{t}=D_{1}e_{t-1}+D_{2}e_{t-2}+\cdots +D_{q}e_{t-q}+Rf_{t}+c_{t},\;t=1,2,\ldots ,T. \end{array}$$

If the lag operator is introduced, it can be expressed as

(4) $$\begin{array}{c} D\left(U\right)e_{t}=-Rf_{t}+c_{t},\;t=1,2,\ldots ,T, \end{array}$$

where *R* can be expressed as

(5) $$\begin{array}{c} R=\left[\begin{array}{cccc} r_{11} & r_{12} & \ldots & r_{1b}\\ r_{21} & r_{22} & \ldots & r_{2b}\\ \ldots & \ldots & \ldots & \ldots \\ r_{m1} & r_{m2} & \ldots & r_{mb} \end{array}\right]. \end{array}$$

Suppose that *e*_*t*_ = (*e*_1*t*_, *e*_2*t*_, ..., *e*_*mt*_)′ represents an *m* dimensional random time series, *t* = 1, 2, ..., *T*, and *e*_*t*_∼*I*(1), that is, corresponding to each data item *e*_*it*_∼*I* (1), *i* = 1, 2, ..., *m*, which is affected by *b* dimensional exogenous time series *f*_*t*_ = (*f*_1*t*_, *f*_2*t*_,…, *f*_*mt*_)′, first, a vector autoregressive model (VAR) is established.

(6) $$\begin{array}{c} e_{t}=D_{1}e_{t-1}+D_{2}e_{t-2}+\cdots +D_{q}e_{t-q}+Rf_{t}+c_{t},\;t=1,2,\ldots ,T. \end{array}$$

If *e*_*t*_ has cointegration relationship, *De*_*t*−1_∼*I*(0) in formula (6) can generate functional relationship.

(7) $$\begin{array}{c} \Delta e_{t}=\eta \phi^{\prime }e_{t-1}-\sum_{i=1}^{m-1}\sum_{j=i+1}^{m}D_{j}\Delta e_{t-i}+c_{t}. \end{array}$$

Among them, *φ′e*_*t*−1_ can be regarded as the error correction term (err_*t*−1_), which reflects the long-term equilibrium relationship between variables, and formula (7) can be rewritten as

(8) $$\begin{array}{c} \Delta e_{t}=\eta {\text{err}}_{t-1}-\sum_{i=1}^{m-1}\sum_{j=i+1}^{m}D_{j}\Delta e_{t-i}+c_{t}. \end{array}$$

The model represented by formula (8) is the vector error correction model (VECM), in which each equation is an error correction model (ECM), and the parameter vector of VECM represents the adjustment speed to the equilibrium state when the equilibrium relationship between variables deviates from the long-term equilibrium state; therefore, this parameter vector is called the adjustment parameter matrix.

The article "Economic Transformation and Security Analysis of RMB Integration Based on CNN" was published in 2022. Journal: Comput Intell Neurosci.

In Figure 2, first, the unit root test is used to test the stability of the daily closing price of currency exchange. If the data are stable, the VAR model is adopted; if the data are not stable, a further cointegration test is carried out on the data; if there is cointegration relationship between the data, the VECM model is adopted; if there is no cointegration relationship between the data, VAR model is adopted. According to the prediction demand, combined with the VAR model and VECM model, set different time prediction spans (42d, 63d, 84d,…). The VAR-VECM model with the best prediction performance is obtained. Based on the residual error of the prediction result of the model, it is used as the input of the convolutional neural network model (CNN), set different time windows and the number of hidden layers, and compare the prediction results of the model under different parameters, so as to obtain the improved CNN (ICNN) model.

In this paper, the ICNN model is used to estimate the equilibrium real exchange rate of RMB. ICNN model defines the equilibrium exchange rate as the final estimate of the exchange rate for the actual effective exchange rate and its related economic fundamental factors through the behavioral relationship established by the econometric method. Specifically, the real effective exchange rate *q* can be expressed as

(9) $$\begin{array}{c} q_{t}=\alpha^{\prime }E_{t}+\beta^{\prime }W_{t}+\gamma^{\prime }B_{t}+\theta_{t}, \end{array}$$

where *B*_*t*_ represents the CNN model, which is used to represent the basic factor vector with long-term impact on the economy, *W*_*t*_ represents the VAR model, which is used to represent the basic factor vector with medium-term impact on the economy, *E*_*t*_ represents the basic factor vector with short-term impact on the economy, *α*, *β*, *γ*, respectively, represent the corresponding coefficient vector, and *θ*_*t*_ represents random interference term.

The article "Economic Transformation and Security Analysis of RMB Integration Based on CNN" was published in 2022. Journal: Comput Intell Neurosci.

The previous empirical studies on equilibrium real exchange rate at home and abroad have a great consensus on the economic fundamentals that affect the real exchange rate. Comprehensive study of the equilibrium exchange rate at home and abroad and the affecting developing (transformation) countries consider external economic fundamentals of the real exchange rate, and we chose the following economic fundamentals: relative labor productivity (XDSCL), foreign trade conditions (TOT), economic openness (OPEN), net worth ratio (NFAR) abroad, government spending ratio (GGR), broad money supply (M2), and RURAL population ratio (RURAL).

Suppose a country USES capital (*K*) and labor (*L*) as two factors of production to produce tradable and nontradable goods. Tradable sector (*T*) and nontradable sector (*N*) exist in the economy, respectively, accounting for the same proportion as foreign countries. *ϑ*1 − *ϑ* tradable goods satisfy the law of one price. The price of tradable goods is determined by the international market, while the price of nontradable goods is determined by the domestic market. Meet the assumption of full employment (limited supply of labor), that is, *L* = *L*_*T*_ + *L*_*N*_. There is a functional relationship between the general price level and the real exchange rate (q rise means the appreciation of the real exchange rate of the country, and the decline means the depreciation); here is to simplify the result; the two departments are drawn as c-d production function*P* = *P*_*T*_^*θ*^ + *P*_*N*_^(1 − *θ*)^*q* = (*P*/*eP*^*∗*^)*Y*_*T*_ = *A*_*T*_*K*_*T*_^*α*^*L*_*T*_^1−*α*^*Y*_*N*_ = *A*_*N*_*K*_*N*_^*β*^*L*_*N*_^1−*β*^. In the optimal case of production, wage is equal to the marginal output of labor, and then,

(10) $$\begin{array}{c} W_{T}=P_{T}*MPL_{T},\\ =P_{T}\left(1-\alpha \right)A_{T}K_{T}^{\alpha }L_{T}^{-\alpha },\\ =\left(1-\alpha \right)P_{T}APL_{T}. \end{array}$$

In the same way,

(11) $$\begin{array}{c} W_{N}=\left(1-\beta \right)P_{N}APL_{N}. \end{array}$$

Since labor can flow freely in a country, wages in the tradable sector and those in the nontradable sector will be equalized. Thus, from (10) and (11),

(12) $$\begin{array}{c} \frac{P_{N}}{P_{T}}=\frac{\left(1-\alpha \right)APL_{T}}{\left(1-\beta \right)APL_{N}},\\ \overset{•}{\left(\frac{P_{N}}{P_{T}}\right)}=\left(1-\alpha \right)\overset{•}{APL_{T}}-\left(1-\beta \right)\overset{•}{APL_{N}}. \end{array}$$

Formula (12) explains that when the labor productivity of a country's tradable sector grows rapidly relative to the domestic nontradable sector, the price of nontradable goods will rise relative to the price of tradable goods, and the internal real exchange rate will appreciate, which is the domestic version of BS effect, and *Ṗ* represents the rate of change of the variable.

The article "Economic Transformation and Security Analysis of RMB Integration Based on CNN" was published in 2022. Journal: Comput Intell Neurosci.

Let the production functions of the two foreign departments be, and the same can be obtained as *Y*_*T*_^*∗*^=*A*_*T*_^*∗*^*K*_*T*_^*∗μ*^*L*_*T*_^*∗*1−*μ*^*Y*_*N*_^*∗*^=*A*_*N*_^*∗*^*K*_*N*_^*∗ν*^*L*_*N*_^*∗*1−*ν*^

(13) $$\begin{array}{c} \frac{P_{N}^{*}}{P_{T}^{*}}=\frac{\left(1-\nu \right)APL_{T}^{*}}{\left(1-\mu \right)APL_{N}^{*}}. \end{array}$$

By combining (12) with (13),

(14) $$\begin{array}{c} \frac{P_{T}^{*}P_{N}}{P_{N}^{*}P_{T}}=\frac{\left(1-\alpha \right)\left(1-\nu \right)APL_{N}^{*}APL_{T}}{\left(1-\beta \right)\left(1-\mu \right)APL_{T}^{*}APL_{N}}. \end{array}$$

When the one price theorem is established, there is the nominal exchange rate of two countries, and then, the real exchange rate q of the country is *e*=(*P*_*T*_/*P*_*T*_^*∗*^)*e*.

(15) $$\begin{array}{c} q=\frac{P}{eP^{*}},\\ =\frac{P_{T}^{\theta }P_{N}^{1-\theta }}{eP_{T}^{*\theta }P_{N}^{*1-\theta }},\\ ={\left[\frac{\left(1-\alpha \right)\left(1-\nu \right)APL_{N}^{*}APL_{T}}{\left(1-\beta \right)\left(1-\mu \right)APL_{T}^{*}APL_{N}}\right]}^{1-\theta },\\ \ln\;q=\left(1-\theta \right)\ln\frac{\left(1-\alpha \right)\left(1-\nu \right)}{\left(1-\beta \right)\left(1-\mu \right)}+\left(1-\theta \right)\ln\frac{\left(APL_{T}/APL_{N}\right)}{\left(APL_{T}^{*}/APL_{N}^{*}\right)},\\ \dot{q}=\left(1-\theta \right)\left[\left(\overset{•}{APL_{T}}-\overset{•}{APL_{N}}\right)-\left(\overset{•}{APL_{T}^{*}}-\overset{•}{APL_{N}^{*}}\right)\right]. \end{array}$$

Formula (15) proves that when a country's tradable sector labor productivity shows a “relative growth,” its external real exchange rate appreciates.

Considering the problem of surplus rural labor in China, the transition from the agricultural population to the manufacturing population will have an important impact on the rise of the wage rate and further restrict the appreciation of the real exchange rate, and this paper introduces the demographic factor into ICNN and sets the following benchmark framework for empirical analysis of the equilibrium exchange rate of RMB.

(16) $$\begin{array}{c} {\text{LICNN}}_{t}=\alpha +\beta_{1}{\text{LXDSCL}}_{t}+\beta_{2}{\text{LTOT}}_{t}+\beta_{3}{\text{LOPEN}}_{t}+\beta_{4}{\text{LNFAR}}_{t}+\beta_{5}\text{LGGR}+\beta_{6}\text{LM}2_{t}+\beta_{7}{\text{RURAL}}_{t}+u_{t}. \end{array}$$

LICNN represents the natural logarithm of the variable of the real effective exchange rate of RMB, and the latter variable is treated in the same way.

The article "Economic Transformation and Security Analysis of RMB Integration Based on CNN" was published in 2022. Journal: Comput Intell Neurosci.

## 3. Empirical Analysis

### 3.1. Data Source and Illustration

As the relative price of currency, the exchange rate serves as the basis for conveying information to the market as a price variable. At the same time, from the perspective of the structural breakpoint in statistical research, the first reform of the RMB exchange rate system on January 1, 1994, resulted in a huge change in the nominal exchange rate, and the statistical results including this breakpoint were lack of robustness. Therefore, this paper chooses 1994 as the starting point of the time series. Given the relatively small number of annual data since 1994, the statistical results are not robust, and quarterly data, which are more frequent than annual data, may contain more important economic information. In order to reduce information leakage and provide sample data of sufficient time series, this paper adopts high-frequency quarterly data. The starting and ending points of samples are the first quarter of 1994 and the third quarter of 2018, respectively, so as to obtain 99 sample points. As the population data only have annual data, it is smoothed quarterly according to the annual growth rate. All data are from the WIND database.

#### 3.1.1. Relative Labor Productivity (XDSCL)

Relative labor productivity is an important basic factor affecting the real exchange rate, and labor productivity affects the real exchange rate through the Balassa–Samuelson effect (BS effect). Due to the special economic background of the economies in transition, there is a surplus labor force in rural areas, which inhibits the growth of wages, thus leading to the weakening of the BS effect. Therefore, the symbol of this variable in the model cannot be determined.

#### 3.1.2. Terms of Trade (TOT)

The term of trade refers to the ratio of a country's export price index to its import price index. Generally speaking, the improvement of a country's terms of trade will lead to the appreciation of its currency and vice versa. However, due to the opposite effects of “income effect” and “substitution effect” on the exchange rate, the sign of this variable in the model cannot be determined.

#### 3.1.3. Economic Openness

The improvement of economic openness means the reduction of trade barriers and the increase of imports, which will promote the growth of imports relative to exports, resulting in the reduction of trade balance. Therefore, the improvement of economic openness will lead to the depreciation of the real exchange rate; that is, the sign of this variable in the model is expected to be negative.

The article "Economic Transformation and Security Analysis of RMB Integration Based on CNN" was published in 2022. Journal: Comput Intell Neurosci.

#### 3.1.4. Foreign Net Assets Ratio (NFAR)

Foreign net assets refer to the difference between a country's foreign assets and its foreign liabilities, which are mainly expressed in the form of foreign exchange reserves and gold. The decline in foreign net assets means that it is necessary to increase the trade surplus to improve the balance of payments, which generally requires the devaluation of the local currency. Moreover, for emerging economies (transition economies), growth requires foreign savings to finance it, and inflows of foreign capital put upward pressure on real exchange rates. Generally speaking, this indicator is expressed as the ratio of a country's net assets abroad to its GDP. Here, we expect the variable to have a positive sign.

#### 3.1.5. Government Expenditure Ratio (GGR)

Generally speaking, the object of government purchasing expenditure is nontradable goods, so when the government expenditure increases, the demand for nontradable goods increases, and the price has upward pressure, and the real exchange rate will appreciate and vice versa. This index is expressed as the ratio of total government expenditure to GDP. The sign for this variable in the model is expected to be positive.

#### 3.1.6. Broad Money Supply (M2)

When the broad money supply M2 expands, the inflation rate will rise, and the current account balance of the country will deteriorate. In this case, the exchange rate depreciation is required to maintain the sustainability of the external balance. Conversely, when M2 contracts, the exchange rate should appreciate. Therefore, the expectation is negatively correlated.

#### 3.1.7. RURAL Population Ratio (RURAL)

Due to China's special urban-rural dual structure, the rural surplus labor force is more prominent than other countries, and there is hidden unemployment in rural areas, so labor force is not full employment. At the same time, due to the factors of structural transformation, in this process, labor force is almost infinite supply within a certain period of time. These factors will restrain the increase in the wage rate to some extent. Only when the surplus labor force is fully released from the countryside, hidden unemployment is reduced to a certain extent, and the labor force is no longer infinite supply, and the key wage transmission mechanism in the BS effect will play its due role. Therefore, the change in China's rural surplus labor force measured by the ratio of rural population variable is expected to be negatively correlated with the real exchange rate.

The article "Economic Transformation and Security Analysis of RMB Integration Based on CNN" was published in 2022. Journal: Comput Intell Neurosci.

Based on the above analysis, we express the theoretical model of the RMB behavioral equilibrium exchange rate as follows:

(17) $$\begin{array}{c} \text{ICNN}=f\left(\overset{?}{\text{XDSCL}},\overset{?}{\text{TOT}},\overset{-}{\text{OPEN}},\overset{+}{\text{NFAR}},\overset{+}{\text{GGR}},\overset{-}{\text{M}2},\overset{-}{\text{RURAL}}\right). \end{array}$$

ICNN stands for the RMB equilibrium exchange rate; XDSCL represents labor productivity; TOT denotes the terms of trade; OPEN denotes openness to the outside world; NFAR represents the ratio of foreign net assets; GGR represents government expenditure ratio; M2 is the broad money supply; RURAL represents the rural population ratio. The sign above the theoretical model expression is the sign of the first partial derivative of each variable, indicating the change direction of the RMB equilibrium exchange rate, namely the theoretical expectation of the change direction of the equilibrium exchange rate, when the basic economic factors increase. The question mark indicates that the relationship between the two cannot be determined temporarily.

### 3.2. The Unit Root Test

First, the stationarity of each sequence was analyzed by the ADF unit root test. The test results are shown in Table 2.

### 3.3. Johansen Cointegration Test

According to the results of the ADF test, the original sequence of all variables is not stable, but the first-order difference sequence is stable, which is the *I*(l) sequence. Therefore, the stationarity of data requires the analysis based on the cointegration framework. Here, the Johansen cointegration test method is adopted for testing.

First, the lag order used in VAR analysis was selected. Considering the data frequency and sample length in this paper, when selecting the maximum lag order of the VAR system, 8 was selected. The VAR(8) system was finally selected according to the AIC criterion in Table 3.

Then, we will examine the rationality of the VAR(8) model. It has been tested that the eigenvalues of the difference equations of the VAR(8) model are all less than 1 and located in the unit circle, which indicates that the VAR(8) system is reasonable, as shown in Figure 3.

Johansen cointegration test is conducted. Trace test and maximum eigenvalue test indicate the existence of 7 and 7 cointegration equations, respectively, indicating the existence of cointegration relations.

Although the maximum eigenvalue statistic indicates that there are 7 cointegration equations, there is only one cointegration equation that contains all variables. The standardized equation is given in Table 4.

The article "Economic Transformation and Security Analysis of RMB Integration Based on CNN" was published in 2022. Journal: Comput Intell Neurosci.

Thus, we can obtain the long-term equilibrium relationship between the real exchange rate of RMB and the economic fundamentals that determine its changes.

(18) $$\begin{array}{c} \text{LICNN LXDSCL}=24.67+0.452+0.496\text{ LTOT }0.321\text{ LOPEN LNFA LGGR }1.201+0.336+0.104\text{ LM}2-0.088*\text{RURAL.} \end{array}$$

As can be seen from Table 3, except for the nonsignificant external net assets, all other variables are significant at the significance level of 5%. This shows that economic fundamentals such as relative labor productivity, terms of foreign trade, openness, government expenditure ratio, broad money supply, and difference equations ratio of difference equations rural population are important medium- and long-term determinants of RMB's real exchange rate.

From the cointegration equation, we can see that all the variable signs that determine the direction are consistent with what we expect. An increase in the ratio of government spending leads to an appreciation of the real exchange rate. An increase in openness, the ratio of difference equations broad money supply to difference equations rural population, would devalue the real exchange rate. The sign of relative labor productivity is positive, indicating that there is a BS effect in the sample period we discussed. The increase in China's relative labor productivity with foreign countries makes the real exchange rate of RMB appreciate. The negative sign of the terms of trade indicates that the substitution effect generated by the improvement of the terms of trade is greater than the income effect, resulting in the depreciation of the real exchange rate.

### 3.4. The Calculation of EER and The Degree of Its Misalignment

The improved convolutional neural network model (ICNN) divides equilibrium exchange rate into short-term equilibrium real exchange rate (CERER) and long-term equilibrium real exchange rate (PERER). It uses cointegration technology to find the relationship between short, medium, and long-term economic factors affecting internal equilibrium and external equilibrium and the real exchange rate in reality and then determines the ERER level of the equilibrium real exchange rate. According to the definition of misalignment of the exchange rate by Williamson [16], misalignment of the real exchange rate refers to the continuous deviation of the real exchange rate from its equilibrium level. Therefore, we can obtain the measure of the dislocation of RMB's real exchange rate.

(19) $$\begin{array}{c} \text{MIS}=\frac{\text{REER}-\text{ERER}}{\text{ERER}}\times 100\%. \end{array}$$

Figure 4 shows the comparison between the real RMB exchange rate REER and the long-term equilibrium real RMB exchange rate PERER based on Johansen cointegration.

The article "Economic Transformation and Security Analysis of RMB Integration Based on CNN" was published in 2022. Journal: Comput Intell Neurosci.

After obtaining the PERER estimate of the RMB long-term equilibrium real exchange rate, we use (19) to measure the long-term dislocation of the RMB real exchange rate.

(20) $$\begin{array}{c} \text{TMIS}=\frac{\text{REER}-\text{PERER}}{\text{PERER}}\times 100\%. \end{array}$$

In the above formula, TMIS represents the long-term dislocation of the real exchange rate, and PERER represents the long-term equilibrium real exchange rate. The long-term dislocation of the real exchange rate of RMB obtained from the (18) measure is shown in Figure 5.

### 3.5. The Analysis of Empirical Results

On the whole, the RMB real exchange rate has experienced four periods of undervaluation and one period of overvaluation. The following detailed analysis of the long-term dislocation of the real exchange rate of the RMB cyclical changes.

Major undervaluation stages are as follows:

1. From the first quarter of 1994 to the third quarter of 1997, the real exchange rate of RMB was undervalued. On January 1, 1994, China implemented the integration of the official exchange rate of RMB with the market price of foreign exchange adjustment. The official exchange rate of RMB depreciated from 5.8 RMB/usd in the previous trading day to 8.7 RMB/usd in that day. The substantial depreciation of the RMB nominal exchange rate resulted in the undervaluation of the RMB real exchange rate in the sample period. Subsequently, the RMB adopted the exchange rate policy of pegging to the US dollar, while the rising domestic price level gradually reduced the degree of RMB's real exchange rate undervaluation.
2. From the third quarter of 1998 to the third quarter of 2001, the real exchange rate of RMB was undervalued. As the Asian financial crisis has receded, Asian currencies have slowly appreciated, and the real exchange rate of the renminbi has fallen. At the same time from 1998, China entered the stage of deflation. In 1998, the year-on-year increase of CPI in China was −0.8%. It was −1.4% in 1999.
3. From the second quarter of 2002 to the first quarter of 2009, the real exchange rate of RMB was undervalued. After 2002, the US dollar continued to depreciate significantly, and the real exchange rate of RMB in China changed from overvaluation to undervaluation. With the second reform of the RMB exchange rate system in July 2005, the peg to the US dollar was changed to a basket of currencies, a managed floating exchange rate system was implemented, and the undervaluation of the RMB real exchange rate began to decrease after reaching the peak at the end of 2005.
4. From the fourth quarter of 2009 to the fourth quarter of 2011, the real exchange rate of RMB was undervalued. With the passing of the inflation peak in 2008, China entered a slight deflation stage in 2009. At the same time, the real exchange rate of RMB also experienced a temporary decline, which made the real exchange rate of RMB gradually become undervalued.

The article "Economic Transformation and Security Analysis of RMB Integration Based on CNN" was published in 2022. Journal: Comput Intell Neurosci.

Major overvaluation stages are as follows:

1. From the fourth quarter of 1997 to the third quarter of 1998, the real exchange rate of RMB was overvalued. Due to the most serious inflation since China's reform and opening up in 1995, the general price level soared sharply, and the real exchange rate converted to the overvaluation stage from 1997 to 1998 and reached the peak in the first quarter of 1998, with an overvaluation of 9.5%. An important factor that caused such a serious misalignment of the RMB's real exchange rate was the Chinese government's commitment not to devalue the RMB during the Asian financial crisis in 1997. Because of the pegging policy of the RMB to the US dollar at that time, the RMB appreciated sharply with the US dollar, resulting in the overvaluation of the RMB real exchange rate.
2. From the third quarter of 2001 to the second quarter of 2002, the real exchange rate of RMB was overvalued. Since 2000, China's economy has gradually stepped out of deflation, and the US dollar began to appreciate sharply from the first quarter of 2000 until 2002 when the real exchange rate of the US dollar rose by a cumulative rate of 8%. These factors make the real exchange rate of RMB overvalued at this stage.
3. From the first quarter of 2009 to the fourth quarter of 2009, the real exchange rate of RMB was overvalued. Affected by the financial crisis in developed countries caused by the subprime crisis in the United States at the end of 2008, China's steady economic growth relative to the western developed countries makes the expectation of RMB appreciation strong.
4. From the fourth quarter of 2011 to the first quarter of 2017, the real exchange rate of RMB was overvalued. With the continuous and steady growth of China's economy and the promotion of economic transformation, the strategies of “going global” and “One Belt And One Road” were successively proposed, and the RMB was planned to be included in the SDR of the IMF. All these require the strong exchange rate.

### 3.6. Further Discussion on RMB Misalignment

Yuan undervalued real exchange rate stage is closely related to China's export-led economic model because there is a great quantity of recessive unemployment in rural China, mainly labor-intensive industries in the early years of the development of the rise of manufacturing can quickly absorb the surplus labour, in order to obtain an export competitive advantage, and the RMB exchange rate level is low. Therefore, from 1994 to 2012, except for a few intermittent overvaluation, the RMB's real exchange rate was basically undervalued. An important supply-side factor that determines the real exchange rate level is the Balassa–Samuelson effect. When using the ICNN model to calculate the exchange rate of emerging market economies, the country characteristics factor is an important consideration in the modeling. Due to the special economic background of China's economies in transition, there is a surplus labor force in rural areas, and the growth of wages is suppressed, which leads to the weakening of the Balassa–Samuelson effect, and then, the real exchange rate is suppressed. After the gradual disappearance of China's demographic dividend and the basic consumption of surplus rural labor force, the rise of the wage rate will be further reflected in the appreciation of the real exchange rate.

The article "Economic Transformation and Security Analysis of RMB Integration Based on CNN" was published in 2022. Journal: Comput Intell Neurosci.

## Figures and Tables

**Figure 1:** (a) Annual growth rate of labor productivity in China and the United States; (b) China-US relative productivity and RMB real effective exchange rate; (c) cumulative index of China's tradable sector labor productivity and cumulative index of China's wage growth.

**Figure 2:** The generation process of improved CNN model.

**Figure 3:** AR root of VAR(8) system.

**Figure 4:** REER of RMB real exchange rate and PERER of RMB long-term equilibrium real exchange rate.

**Figure 5:** The long-term dislocation of RMB real exchange rate based on ICNN.

**Table 1:** Problems of traditional analysis methods.

Traditional analysis method	Specific definition	Existing problems
Event-driven analysis	Through the analysis of macroeconomic events and major events that can affect the development of enterprises, make judgments that may have an impact on the future, so as to predict the trend of the financial market.	Investors should always pay attention to the market and be close to the market, so as to obtain information quickly and accurately; investment is excessively dependent on a certain entity, and if only a few people are optimistic about it, they will not be able to make profits or even losses.

Performance-driven analysis	Taking the performance of the sustainable development of the enterprise as the consideration, by comprehensive consideration of the industry, products, management mode, financial status, and other conditions of the enterprise, judge the future development direction and performance expectation of the enterprise, so as to predict the trend of the financial market.	It is necessary to grasp the performance report of the company at all times and comprehensively consider all indicators of the company, so as to predict the future performance of the company; the selection of companies and the number of companies have an important impact on the accuracy of financial market assessment, and if the number of companies is small and unrepresentative, judgment errors will occur.

The article "Economic Transformation and Security Analysis of RMB Integration Based on CNN" was published in 2022. Journal: Comput Intell Neurosci.

**Table 2:** ADF test results of the stationarity of each variable.

Variable	Test form (*c*, *t*, *l*)	The ADF statistics	*P* values	Stationarity
LREER	(*c*, *t*, 0)	2.27	0.45	Not smooth
ΔLREER	(*c*, 0, 0)	8.58	0	Smooth^*∗∗∗*^
LXDSCL	(*c*, *t*, 0)	1.21	0.90	Not smooth
ΔLXDSCL	(*c*, 0, 0)	9.58	0	^*∗∗∗*^
LTOT	(*c*, *t*, 0)	3.96	0.01	Not smooth
ΔLTOT	(*c*, 0, 0)	10.57	0	^*∗∗∗*^
LOPEN	(*c*, *t*, 0)	1.11	0.92	Not smooth
ΔLOPEN	(*c*, 0, 0)	9.99	0	^*∗∗∗*^
LNFA	(*c*, *t*, 2)	0.81	0.99	Not smooth
^Δ^ The NFA	(*c*, 0, 1)	4.01	0	^*∗∗∗*^
LGGR	(*c*, *t*, 3)	0.94	0.95	Not smooth
ΔLGGR	(*c*, 0, 2)	20.15	0	^*∗∗∗*^
LM2	(*c*, 0, 0)	1.40	0.86	Not smooth
^Δ^M2	(*c*, 0, 0)	6.93	0	^*∗∗∗*^
The RURAL	(*c*, *t*, 1)	2.75	0.22	Not smooth
^Δ^The RURAL	(*c*, 0, 0)	3.60	0	^*∗∗∗*^

**Table 3:** VAR lag order selection criteria.

Lag	LogL	LR	FPE	AIC	SC	HQ
1	1496.404	NA	2.95*e* − 24	31.48140	29.71552^*∗*^	30.76898^*∗*^
2	1570.221	121.6765	2.44*e* − 24	31.69716	28.16540	30.27231
3	1641.096	104.3656	2.25*e* − 24	31.84826	26.55062	29.71099
4	1735.815	122.8231^*∗*^	1.33*e* − 24^*∗*^	32.52342	25.45990	29.67373
5	1797.433	69.06545	1.83*e* − 24	32.47105	23.64165	28.90894
6	1856.515	55.83608	3.14*e* − 24	32.36297	21.76769	28.08843
7	1932.755	58.64593	4.77*e* − 24	32.63197	20.27082	27.64502
8	2040.066	63.67940	5.49*e* − 24	33.58387^*∗*^	19.45684	27.88450

**Table 4:** Standardized equations of cointegration test.

LREER	LXDSCL	LTOT	LOPEN	LNFA	LGGR	LM2	RURAL	C
1.0000	0.452	0.496	0.321	0.104	0.336	1.201	0.089	24.67
The standard deviation	0.250	0.237	0.171	0.152	0.194	0.529	0.055	
*T* value	1.807	2.097	1.873	0.686	1.735	2.271	1.618	
Logarithmic likelihood ratio	1918.85							

## Data Availability

The dataset used in this paper is available from the corresponding author upon request.
